This article has been retracted.

# *Pseudomonas aeruginosa* mucinous phenotypes and *algUmucABD* operon mutant characteristics obtained from inpatients with bronchiectasis and their correlation with acute aggravation

**DOI:** 10.3389/fcimb.2024.1402348

**Published:** 2024-07-29

**Authors:** Yuxue Tan, Zhongshang Dai

**Affiliations:** ^1^ Department of Internal Medicine, The First People’s Hospital of Fuquan City, Fuquan, Guizhou, , China; ^2^ Department of Infectious Diseases, The Second Xiangya Hospital, Central South University, Changsha, Hunan, China

**Keywords:** bronchiectasis, *Pseudomonas aeruginosa*, gene mutations, *algUmucABD/algTmucABD* operon, acute exacerbations

## Abstract

**Objective:**

Although the mechanism is unclear, *Pseudomonas aeruginosa* (PA) infection directly affects the frequency of acute exacerbations in patients with bronchiectasis. The aims of this article are to analyze the genetic mutation characteristics of the *algUmucABD* operon in PA, isolated from hospitalized patients with bronchiectasis, and to explore independent risk factors for frequent acute exacerbations of bronchiectasis.

**Methods:**

Based on the number of acute exacerbations that occurred in the past year, these patients with bronchiectasis were divided into those with frequent acute exacerbations (Group A) and those with non-frequent acute exacerbations (Group B). We identified the distribution of mucoid phenotypes (MPs) and alginate morphotypes (AMs) in PA, and classified them into I–IV categories based on their different AMs; otherwise, the gene mutation types (GMTs) of the *algUmucABD* operon were tested. Subsequently, the relationship between GMT, MP, and AM and the independent risk factors for frequent acute exacerbations in patients with bronchiectasis were explored.

**Results:**

A total of 93 patients and 75 PA strains, from January 2019 to August 2023, were included in this study. The MP and AM distributions of PA were as follows: 64 strains (85.33%) of mucoid (the AMs were 38 strains of type I, 3 strains of type II, and 23 strains of type IV) and 11 strains of non-mucoid (the AM was type III only). Mucoid PA with *algU*, *mucA*, *mucB*, and *mucD* mutations accounted for 19.61%, 74.51%, 31.37%, and 50.98%, respectively. GMT was divided into the following: *mucA* mutations only, *mucA* combined with other gene mutations, other gene mutations without *mucA* mutations, and without gene mutations. In 91.7% of PA with type I of AM, only *mucA* mutations occurred, and in both separate MP and AM, the GMT differences were statistically significant. Lastly, the number of lung lobes with bronchiectasis and the number of PA with *mucA* mutations only were the independent risk factors for frequent acute exacerbations.

**Conclusion:**

The *mucA* mutation was primarily responsible for the mucoid of MP and type I of AM in PA, and it was also an independent risk factor for frequent exacerbations of bronchiectasis.

## Introduction

*Pseudomonas aeruginosa* (PA) is a member of the conditionally pathogenic bacterial group that frequently causes nosocomial infections, including pneumonia associated with ventilators and acute exacerbations of illnesses in patients with impaired immune systems (Diggle and Whiteley, 2020). One of the main virulence factors of PA during respiratory infections is the extracellular matrix found in biofilms, which includes proteins, extracellular DNA, and polysaccharides (Malhotra et al., 2019; Jurado-Martín et al., 2021). Extracellular polysaccharides, such as Psl/Pel and alginate, are important for adhesion, scaffolding, and stabilizing biofilms, but they also have different protective roles: Psl mainly resists immune cell action, Pel resists antibiotic treatment, and alginate shields the biofilm from unfavorable environments like oxidative stress formed during cell phagocytosis (Pang et al., 2019; Karygianni et al., 2020).

Studies have shown that 4 days after PA infection, wild-type strains begin to synthesize alginate from non-mucoid to mucoid type, thereby mediating stable attachment. Then, a large amount of alginate synthesis can promote the maturation of biofilm and the formation of microcolonies; alginate also plays an important role in the dispersion of colonies in the later stage, and the result is a vicious cycle (Hay et al., 2009a; Goltermann and Tolker-Nielsen, 2017; Alcaraz-Serrano et al., 2019). The mucoid phenotypes (MPs) of PA can be roughly divided into mucoid and non-mucoid, but it has been found that PA manifests as inconsistent alginate morphotypes (AMs) depending on the degree of alginate synthesis. Thus, AM is a further classification of the PA phenotypes; however, there is a lack of relevant research (Damron and Yu, 2011; Delgado et al., 2018; Cross et al., 2020).

Bronchiectasis (hereafter referred to as non-cystic fibrosis bronchiectasis) is typified by a vicious cycle of “infection–inflammation–airway remodeling–disruption of lung function and impaired clearance–bacterial colonization” (McShane et al., 2013; Flume et al., 2018). Approximately 25%–50% of patients with bronchiectasis are infected with PA, and national and international studies have shown that PA is one of the main causative organisms in the stabilization and acute exacerbation phases of patients with bronchiectasis (Tunney et al., 2013; Lin et al., 2016; Chalmers et al., 2018; Chandrasekaran et al., 2018; Dhand, 2018). In contrast to other prognostic indicators (frequency of acute exacerbations, hospitalization, and quality of life), Chai et al (Chai and Xu, 2020). observed that PA was only an independent risk factor for mortality in patients with frequent acute exacerbations (twice or more per year).

By comparing the clinical features, MP and AM distributions, and *algUmucABD* operon mutation profiles of PA between patients with frequent and infrequent acute exacerbations, the study aimed to analyze the independent risk factors for frequent exacerbations of bronchiectasis and offer some insights into the treatment of patients with bronchiectasis with PA infections.

## Materials and methods

This study focused on the inpatients with bronchiectasis with PA infection and the PA strains isolated from these patients at Guizhou Provincial People’s Hospital in China between January 2019 and August 2023. The study was approved by the Guizhou Provincial People’s Hospital Ethics Committee (Approval No. 2021207). We obtained informed consent from all study patients.

### Study patients

All patients were diagnosed with bronchiectasis based on Quint et al.’s diagnostic criteria (Quint and Smith, 2019; Bronchiectasis Expert Consensus Writing Group and Pulmonary Infection Assembly, Chinese Thoracic Society, 2021). The condition is primarily identified by high-resolution computed tomography (HRCT) of the chest demonstrating columnar or cystic bronchiectasis. We included in the study patients who were ≥18 years of age and ever had PA isolated from lower respiratory tract specimens (sputum or alveolar lavage fluid), regardless of comorbidities with other pathogenic bacterial infections and initiation of antibiotic therapy; among them, those who had undergone surgeries such as solid organ and bone marrow transplants, were treated with immunosuppressive drugs, suffered from malignancy, or had neurological disorders and/or psychiatric disorders in the last 6 months were excluded (Alcaraz-Serrano et al., 2019).

Combining the definitions of acute exacerbation and frequent acute exacerbation (acute exacerbations ≥2/year) of bronchiectasis in the Saudi Thoracic Society guidelines (Al-Jahdali et al., 2017) and the Chinese Expert Consensus on the Diagnosis and Treatment of Bronchiectasis in Adults (Bronchiectasis Expert Consensus Writing Group and Pulmonary Infection Assembly, Chinese Thoracic Society, 2021), the patients were classified into those with frequent acute exacerbations (Group A) and those with non-frequent acute exacerbations (Group B). The following data were collected from these patients: (1) basic information: medical record number, gender, age, length of hospitalization, body mass index (BMI), comorbidities, and discharge diagnosis; (2) medical history: history of smoking and the number of bronchiectasis-related hospitalizations and acute exacerbations in the last 1 year; (3) investigations: thoracic HRCT and pulmonary function; (4) laboratory data (all results of the first test after the patient’s admission to the hospital), including white blood cell (WBC), neutrophil percentage (N%), C-reactive protein (CRP), and albumin; and (5) the degree of dyspnea at admission, which was assessed using the Modified Medical Research Council scale (mMRC).

### Analysis of mucinous phenotypes and *algUmucABD* operon mutant characteristics of PA strains

PA was isolated from patients’ lower respiratory tract specimen and cultured using Columbia blood agar and chocolate agar media, and the MP and AM of PA were characterized using Luria–Bertani (LB) and *Pseudomonas* isolation agar (PIA) plates. AM was classified into types I–IV according to the mucoid transformation of the strains on both LB and PIA media: type I: obvious mucoid transformation on both media; type II: mucoid transformation only on PIA medium; type III: non-mucoid transformation on both media; type IV: non-mucoid transformation was observed on 1–3 days of incubation, and very slight but observable mucoid transformation on both media after prolonged incubation to 4–7 days (Ciofu et al., 2008). Types I, II, and IV in AM were defined as mucoid and type III was defined as non-mucoid; meanwhile, mucoid and non-mucoid were defined as MP (PAO1 was used as the quality control organism). Simultaneously, we analyzed the mutant profiles of the *algUmucABD* operon (see the **Appendix** for this part of experiment).

### Statistical analysis

The data were analyzed using Statistical Package for Social Sciences (SPSS) version 23.0 (Armonk, New York, USA). The measurement data were analyzed using the Kolmogorov–Smirnov and the Mann–Whitney *U* tests, and the results were expressed as medians [interquartile range (IQR)] and *Z*-values. Comparisons of dichotomous variables were made using the four-cell table *χ* ^2^ test, with the continuous correction method when there was a cell with a minimum theoretical frequency (*T*_min_) greater than or equal to 1 as well as less than 5; comparisons of multi-categorical variables were made using the row-by-row list *χ* ^2^ test, and Fisher’s exact probability method was chosen when *T*_min_ < 1 or more than 1/5 of the cells had a 1 ≤ *T*_min_ < 5; the results were expressed as numbers (percentages) and *χ* ^2^ values. Graphing was carried out with GraphPad Prism 6.0 (GraphPad Software, USA), Adobe Illustrator CC (Adobe, USA), and Photoshop CC (Adobe, USA). Statistical significance was set at *p* < 0.05.

## Results

### Clinical characteristics of the patients

A total of 108 patients and 92 strains of PA were collected in this study, a total of 15 cases and 17 strains of PA (2 strains were isolated from each of the 2 patients) isolated from them were excluded due to incomplete medical records of patients, and 93 cases and 75 strains of PA were finally included. Specimens were not collected from 18 patients, resulting in a lower number of PA strains than cases.

According to whether the number of exacerbations was greater than or equal to 2 in the last 1 year, 93 patients were divided into those with frequent acute exacerbations (Group A, 47 cases) and those with non-frequent acute exacerbations (Group B, 46 cases) (Bronchiectasis Expert Consensus Writing Group and Pulmonary Infection Assembly, Chinese Thoracic Society, 2021). The comparison found more severe bronchiectasis lesions in Group A (*p* = 0.002) (**Table 1**).

**Table 1:** Analysis of clinical characteristics between Group A and Group B.

Items	Group A	Group B	Statistics	*p*
Total number, *n* (%)	47 (50.5%)	46 (49.5%)		
Female, *n* (%)	22 (46.8%)	23 (50.0%)	0.095	0.758
Age (years)^*^	63 (16.0)	64 (18.0)	−0.073	0.942
*BMI* (kg/m^2^) ^*^	19.5 (4.7)	20.2 (4.4)	−0.742	0.458
Length of hospitalization (days)^*^	9 (5.0)	11 (8.5)	−1.353	0.176
Smoking history, yes, *n* (%)	15 (31.9%)	13 (28.3%)	0.148	0.701
Respiratory failure, yes, *n* (%)	16 (34.0%)	10 (21.7%)	1.747	0.186
The number of hospitalizations in the last 1 year (times) ^*^	2(2)	1 (1)	−4.500	0.000
The number of acute exacerbations in the last 1 year (times) ^*^	3(1)	1 (1)	−7.313	0.000
The number of lungs with bronchiectasis on *HRCT* (lobes)^*^	4 (1)	3.5 (2)	−3.109	0.002
*mMRC*, *n* (%)			0.788	0.852
Grade 0–I	15 (31.9%)	18 (39.1%)		
Grade II	11 (23.4%)	11 (23.9%)		
Grade III	10 (21.3%)	9 (19.6%)		
Grade IV	11 (23.4%)	8 (17.4%)		
Laboratory data				
WBC (×10^9^/L) ^*^	8.3 (5.7)	7.1 (3.2)	−2.106	0.035
N% ^*^	73.7 (18.1)	70.8 (14.3)	−0.957	0.339
CRP (mg/L) ^*^	17.4 (36.0)	15.2 (43.7)	−0.096	0.923
Albumin (g/L) ^*^	35.9 (6.8)	35.7 (8.0)	−0.438	0.661
Comorbidity, *n* (%)				
COPD	29 (61.7%)	23 (50.0%)	1.291	0.256
Asthma	7 (14.9%)	5 (10.9%)	0.335	0.563
Hypertension	12 (25.5%)	14 (30.4%)	0.277	0.598
Diabetes mellitus	9 (19.1%)	6 (13.0%)	0.641	0.423

BMI, body mass index; HRCT, high-resolution computed tomography; mMRC, Modified Medical Research Council; WBC, white blood cell; N, neutrophils; CRP, C-reactive protein; COPD, chronic obstructive pulmonary disease. *Non-normally distributed data and data are shown as median [interquartile range (IQR)].

### The MP and AM of PA

Among the 75 strains of PA, 64 mucoid strains (accounting for 85.33%, with 38 strains of type I, 3 strains of type II, and 23 strains of type IV AM) and 11 non-mucoid strains (with all strains of type III AM) were identified (**Figure 1**).

**Figure 1:** Identification of PA alginate morphotypes on LB and PIA media. Type I: On both media, there was a clear mucoid transition; Types II and III indicate that mucoid transformation was only seen on PIA and not on LB, or that there was no mucoid transformation on either medium.  Type IV: After 1–3 days of incubation, no mucoid transformation was seen; after 4–7 days, there was a very mild but noticeable transformation on both media.

### The mutation sites of various genes in the *algUmucABD* operon and their distribution in the MP

We performed sequencing analysis of *algU*, *mucA*, *mucB*, and *mucD* in the *algUmucABD* operon of the PA strains; gene mutations (referred to as righteous mutations) were detected in 76% of PA (51 mucoid strains and 6 non-mucoid strains). Mucoid strains mutated mainly in *mucA* and *mucD*, while non-mucoid strains mutated mainly in *mucB* and *mucD*. The proportion of PA with *mucA* mutations in mucoid and non-mucoid strains were 59.38% (38/64 strains) and 9.1% (1/11 strains), respectively, with large fragment base deletions and multi-site base insertions being the main causes, while the number of PA with *algU*, *mucB*, and *mucD* gene mutations was 10 (all of which were mucoid), 19 (mucoid 16, non-mucoid 3), and 31 (mucoid 26, non-mucoid 5), respectively, all of which were more common with base-based point mutations. Interestingly, six mutant strains were non-mucoid and 13 non-mutants were mucoid among all of them (the mutations of various genes in the *algUmucABD* operon of 75 PA strains are shown in **Appendix Tables 4**–**7**).

### The GMT of *algUmucABD* operon

According to the mutations of each gene in the *algUmucABD* operon of each PA, 75 PA strains were divided into the following gene mutation types (GMTs): *mucA* mutations only (12 strains); *mucA* merge mutations (26 strains, namely, 14 strains of *mucA* + *mucD*, 2 strains of *mucA* + *mucB*, 5 strains of *mucA* + *algU*, 2 strains of *mucA* + *mucB* + *algU*, 1 strain of *mucA* + *mucB* + *mucD*, and 2 strains of *mucA* + *algU* + *mucB* + *mucD*); other types of gene mutations without *mucA* mutations (19 strains, namely, 4 strains of *mucB*, 7 strains of *mucD*, 7 strains of *mucB* + *mucD*, and 1 strain of *mucD* + *algU*); and no genetic mutation (18 strains).

### The distribution of GMT in the MP and AM

Further comparison revealed statistically significant differences between different GMTs in mucoid and non-mucoid PA (*χ* ^2^ = 9.102, *p* = 0.017) (**Table 2**), and it can be seen that all PA strains, with *mucA* mutations only, were mucoid. In addition, 79.7% of the mucoid PA (mPA) had gene mutations, and 45.5% of the non-mucoid PA had other types of mutations but *mucA*.

**Table 2:** Comparing the various GMTs of PA that are mucoid and those that are not (*n* = 75).

	Mucoid (*n* = 64)	Non-mucoid (*n* = 11)	*χ* ^2^	*p*
GMT, *n* (%)			9.102	0.017
*mucA* mutations only	12 (18.8)	0 (0.0)		
*mucA* merge mutations^★^	26 (40.6)	1 (9.0)		
Other types of mutations^◆^	13 (20.3)	5 (45.5)		
No genetic mutation	13 (20.3)	5 (45.5)		

^★^Including *mucA* + *mucD*, *mucA* + *mucB*, *mucA* + *algU*, *mucA* + *mucB* + *algU*, *mucA* + *mucB* + *mucD*, and *mucA* + *algU* + *mucB* + *mucD*; ^◆^ including *mucB*, *mucD*, *mucB* + *mucD*, and *mucD* + *algU*.

The total number of mutation types for each gene in *algUmucABD* operon, distributed in PA of different AMs, was as follows: *algU* 16 types, *mucA* 32 types, *mucB* 14 types, and *mucD* 28 types in AM type I; only 1 type of mutation was discovered in *algU* and *mucA* in AM type II; then, *mucA* 2 types, *mucB* 4 types, and *mucD* 5 types were discovered in AM type III; and *algU* 5 types, *mucA* 15 types, *mucB* 8 types, and *mucD* 15 types were discovered in AM type IV; their proportions are shown in **Figure 2**.

**Figure 2:** The overall percentage of mutations found in each gene inside the *algUmucABD* operon in PA with various AMs.

Interestingly, we found that 91.7% of strains with *mucA* mutations only exhibited type I AM, the distribution of GMT in other types of AM had no obvious characteristics, and the differences in the distribution of GMT among different AMs were statistically significant (*χ* ^2^ = 23.216, *p* = 0.006) (**Table 3**).

**Table 3:** Comparing the GMT among different AMs of PA (*n* = 75).

	Type I	Type II	Type III	Type IV	*χ* ^2^	*p*
GMT, *n* (%)					23.216	0.006
*mucA* mutations only	11 (91.7) ^αβγ^	0 (0.0)	0 (0.0) ^αβ^	1 (8.3)		
*mucA* merge mutations^★^	15 (55.6)	1 (3.7)	1 (3.7) ^αβ^	10 (37.0)		
Other types of mutations^◆^	6 (33.3)	0 (0.0)	5 (27.8)	7 (38.9)		
No genetic mutation	6 (33.3)	2 (11.1)	5 (27.8)	5 (27.8)		

^α^compared with the group with other types of mutations *p* < 0.05; ^β^compared with the group without mutations p < 0.05; ^γ^compared with the group with mucA merge mutations *p* < 0.05. ^★^Including *mucA* + *mucD*, *mucA* + *mucB*, *mucA* + *algU*, *mucA* + *mucB* + *algU*, *mucA* + *mucB* + *mucD*, and *mucA* + *algU* + *mucB* + *mucD*; ^◆^including *mucB*, *mucD*, *mucB* + *mucD*, and *mucD* + *algU*.

### Risk factors for frequent acute exacerbations of bronchiectasis

First, we compared the MP of PA in patients between Groups A and B and came to the conclusion that the difference was not statistically significant. When we looked at the AM of PA between the two groups, we were surprised to find that the difference was statistically significant and that the percentage of mPA with AM of type I was higher in Group A while the percentage of mPA with AM of type IV was higher in Group B. This finding perfectly explains the immediate reason for the lack of a significant difference in MP between the two groups (**Table 4**).

**Table 4:** Analysis of the distribution of the MP and the AM, the mutation characteristics of the *algUmucABD* operon, in PA between Groups A and B.

	Group A (*n* = 42)	Group B (*n* = 33)	*χ* ^2^	*p*
Mucinous phenotypes, *n* (%)			0.188	0.664
Mucoid	37 (88.1)	27 (81.8)		
Non-mucoid	5 (11.9)	6 (18.2)		
Alginate morphotypes, *n* (%)			8.374	0.029
Type I	27 (64.3) ^α^	11 (33.3)		
Type II	2 (4.8)	1 (3.0)		
Type III	5 (11.9)	6 (18.2)		
Type IV	8 (19.0) ^α^	15 (45.5)		
Genetic mutations, *n* (%)				
*algU* mutants	6 (14.3)	4 (12.1)	0.000	1.000
*mucA* mutants	27 (64.3)	12 (36.4)	5.772	0.016
*mucB* mutants	8 (19.0)	11 (33.3)	1.994	0.158
*mucD* mutants	14 (33.3)	17 (51.5)	2.519	0.112
GMT, *n* (%)			9.426	0.024
*mucA* mutations only	11 (26.2) ^α^	1 (3.0)		
*mucA* merge mutations^★^	16 (38.1)	11 (33.3)		
Other types of mutations^◆^	7 (16.7)	11 (33.3)		
No genetic mutation	8 (19.0)	10 (30.3)		

^α^Compared with group B, p < 0.05. ^★^Including *mucA* + *mucD*, *mucA* + *mucB*, *mucA* + *algU*, *mucA* + *mucB* + *algU*, *mucA* + *mucB* + *mucD*, and *mucA* + *algU* + *mucB* + *mucD*; ^◆^including *mucB*, *mucD*, *mucB* + *mucD*, and *mucD* + *algU*. GMT, gene mutation type.

Analysis of the *algUmucABD* operon mutations in PA revealed that Group A had a larger percentage of PA with *mucA* mutations only than Group B. Nonetheless, there was no discernible difference in the percentage of PA with other GMTs between the two groups (**Table 4**).

### Regression analysis of independent risk factors for frequent acute exacerbations of bronchiectasis

Independent variables included in the binary logistic regression model included patients’ clinical characteristics (BMI, number of lung lobes with bronchiectasis on HRCT, WBC, N%, and etiology) and strain factors (AM, *mucA* mutants, and GMT). The results showed that the number of lung lobes with bronchiectasis on HRCT [OR (95% CI): 1.835 (1.124–2.997), *p* = 0.015] and the *mucA* mutations only in GMT [OR (95% CI): 17.522 (1.806–169.991), *p* = 0.014] were the independent risk factors for frequent exacerbations of bronchiectasis (**Figure 3**).

**Figure 3:** Regression analysis of independent risk factors for frequent acute exacerbations of bronchiectasis. BMI, body mass index; HRCT, high-resolution computed tomography; WBC, white blood cell; N, neutrophils; COPD, chronic obstructive pulmonary disease; CTD, connective tissue disease; ABPA, allergic bronchopulmonary aspergillosis; AMs, alginate morphotypes; GMTs, gene mutation types.

## Discussion

In this experiment, both type I and type IV AMs were classified as mucoid; the difference in MP of PA between Groups A and B was not statistically significant, most likely because Group B had a higher prevalence of type IV but a lower prevalence of type I than Group A. Furthermore, the distribution of strains with *mucA* mutations only in Group A is significantly higher than that in Group B. In the end, the number of lung lobes with bronchiectasis on *HRCT* and PA with *mucA* mutations only, were the independent risk factors for frequent acute exacerbations of bronchiectasis.

The term “mucinous transformation” describes the development of a thick coating of mucus-like material on the surface of the strain as a result of excessive alginate production. The correlation between mucinous transformation and alginate quantification is not well understood (Ciofu et al., 2008). The results indicate that there was a strong correlation between the levels of alginate production measured by overnight incubation in beef broth and the phenotypic characterization of alginate production (types I, II, III, and IV) as determined by the morphology of colonies on PIA and LB plates. The *M* (*Q*_1_, *Q*_3_) of alginate production measured in isolates presenting types I, II, III, and IV, respectively, were 180.69 (16.8–757.9), 79.6 (1.07–449), 0 (0–27.9), and 2 (0–496) mg/L, with statistically significant differences between different groups (Ciofu et al., 2008). This implies that the strain’s synthesis of alginate in a rich medium (such as beef broth) is correlated with the colony shape on PIA plates. Our study yielded a detection rate of 85.33% of mucoid strains, which is correspondingly higher than other studies that determined the strains with AM of types II and IV to be the non-MP (Ciofu et al., 2008; Candido Caçador et al., 2018). Furthermore, strains exhibiting mutations in *mucB* and/or *mucD* after extended incubation on particular media are thought to be the cause of type II and type IV of AM. As a result, it has been reported that clinical microbiology laboratories frequently misidentify this class of PA isolates as non-mucoid (Ciofu et al., 2008).

This study found that the high amount of alginate synthesis by PA was closely linked to the mutations in *mucA* and *mucD*. This phenomenon does not fully align with findings documented in other academic publications (Bragonzi et al., 2006; Pulcrano et al., 2012), whereby *mucA* mutation was identified as the primary cause, and the following are some potential explanations for this: First, as was previously indicated, the mucoid strains included both *mucA* and *mucD* mutations that were present in type I and type IV strains. Additionally, the methodology used to determine mPA in this study differed from that used in previous investigations. Second, there is no pertinent additional literature for this analysis, and 71.43% of the mPA in our study have other types of mutations, except for *mucA* mutations. Lastly, the bulk of PA cases documented in the literature came from patients with cystic fibrosis (CF). This is likely because the lung microenvironments of people with these two illnesses select for PA strains in distinct ways. This theory needs to be tested via more research (Boucher et al., 1997; Anthony et al., 2002; Bragonzi et al., 2006; Ciofu et al., 2008; Meng et al., 2009; Moyano and Smania, 2009; Ciofu et al., 2010; Pulcrano et al., 2012; Candido Caçador et al., 2018; Chandrasekaran et al., 2018; Liu et al., 2022). Interestingly, we found that the strains with *algU* mutations were all mucoid; however, other studies have found that 30%–55% of non-mPA isolated from patients with CF were reversed strains, as they had mutations in both *mucA* and *algU*, and the strains with *algU* mutations were almost non-mucoid (Ciofu et al., 2008; Sautter et al., 2012; Candido Caçador et al., 2018). It has also been pointed out the *algU* mutation is the most common mechanism of reversal in non-mucoid strains (DeVries and Ohman, 1994; Schurr et al., 1994), but this mechanism is not dependent on *algU* because *algB*, *algR*, and *algU* together are important regulators of alginate synthesis, and therefore, *algB* and *algR* mutations may be a potential mechanism of reversal (Sautter et al., 2012). It is believed that none of the mutations found in *algU* in this study might alter the function of AlgU or that other regulatory mechanisms that we are not yet aware of may be at play in the five PA strains that exhibited both *mucA* and *algU* mutations and were all mucoid.

We found that 91.7% of PA with AM type I had *mucA* mutations only, suggesting that *mucA* mutations are the main mechanism for AM of type I. In addition to *mucA* mutations, PA with other gene mutations showed type I, type III, and type IV, and strains with no mutations had a distribution of all four AMs. Therefore, we hypothesized that, in addition to the *algUmucABD* operon, alginate biosynthesis is also affected by other regulatory mechanisms. Post-translational regulation of alginate is regulated by factors such as bis-(3′-5′)-cyclic dimeric guanosine monophosphate (c-di-GMP), Alg44-Alg8 complex, AlgE, and AlgC, which are essential for alginate polymerization and secretion (Oglesby et al., 2008; Hay et al., 2009b). It is still unclear what the specific environmental signals that induce alginate production are and how to detect the mechanisms behind them (Hay et al., 2014), as well as the regulatory mechanisms between the regulators (e.g., *algU*, AmrZ, and c-di-GMP) and the signals. It is possible that overexpression or inactivation of some of these regulators could have a significant impact on the polymerization and secretion of the alginate (Hay et al., 2014).

Because of the concurrence of multi-gene mutations in the *algUmucABD* operon of the same PA strain, different gene mutations that occurred in the same strain were defined as one kind of mutation type, and then all of the mutation types were categorized into four GMTs based on whether there were mutations, whether with *mucA* mutations, and further whether with *mucA* mutations only. Comparing the differences between PA with different GMTs in Groups A and B, we found that PA with *mucA* mutations only were more frequent in Group A, whereas the differences between PA with other GMTs were not statistically significant. Further regression analysis showed that the proportion of PA with *mucA* mutations only [OR (95% CI): 17.522 (1.806–169.991), *p* = 0.014] was an independent risk factor for frequent exacerbations of bronchiectasis; i.e., the risk of frequent exacerbations in patients with *mucA* mutations of the *algUmucABD* operon was 17.522 times higher than that of patients with no mutations. The relationship between *mucA* mutations and the prognosis of patients with bronchiectasis is currently unknown, and the studies have reported that *mucA* mutations were an independent risk factor for death in patients with COPD [OR (95% CI): 10.43 (1.53–70.90), *p* = 0.017] (Jung et al., 2018).

Additionally, current alginate solubilizers for PA super mucinous biofilm can only disrupt the microcolony structure, and the effect on mucinous biofilm alginate is minimal and for unknown reasons (Hay et al., 2009a; Hay et al., 2009b). This study concluded that PA infections, along with *mucA* mutations, increase the risk of frequent exacerbations of bronchiectasis by 16.52-fold. Therefore, drugs that can block or reverse *mucA* mutations will be a crucial breakthrough in the clinical treatment of PA chronic infections. In addition, early and effective eradication therapy in the early stages of PA infection (antecedent to *mucA* mutations) may be essential to improve the prognosis of patients with bronchiectasis.

This study has some shortcomings. First of all, the number of collected bronchiectasis medical records and PA strains was small, comprising inpatients only and excluding ambulatory patients with relatively stable conditions, which may limit the generalizability of the results of this study to all patients with bronchiectasis. It is necessary to do a large-scale multicenter study at a later stage. Secondly, some patients had already started antibiotic therapy at the time of inclusion in the study; thus, the effect of antibiotic use on the MP, AM, and the mutational characteristics of the *algUmucABD* operon cannot be evaluated. The median length of hospitalization for all patients was 10 days, which is relatively short compared with the median bronchiectasis history (10 years); thus, the use of antibiotics within a short period of time after hospitalization had a relatively small impact on the above factors; on the other hand, a history of prolonged out-of-hospital antibiotics use in most patients made it difficult to control the factor of antibiotic use.

## Data availability statement

The original contributions presented in the study are publicly available. This data can be found here: https://nmdc.cn/accession: SUB1720353200260.

## Ethics statement

The studies involving humans were approved by the Guizhou Provincial People’s Hospital Ethics Committee (Approval No. 2021207). The studies were conducted in accordance with the local legislation and institutional requirements. The participants provided their written informed consent to participate in this study.

## Author contributions

YT: Conceptualization, Data curation, Formal analysis, Investigation, Methodology, Project administration, Resources, Writing – original draft, Writing – review & editing, Validation, Visualization. ZD: Conceptualization, Data curation, Methodology, Supervision, Validation, Visualization, Writing – review & editing, Project administration.
